# Anatomical Phase Extraction (APE) Method: A Novel Method to Correct Detrimental Effects of Tissue-Inhomogeneity in Referenceless MR Thermometry—Preliminary Ex Vivo Investigation

**DOI:** 10.1155/2021/5566775

**Published:** 2021-08-10

**Authors:** Chien-Feng Judith Huang, Win-Li Lin, San-Chao Hwang, Ching Yao, Hsu Chang, Li-Wei Kuo

**Affiliations:** ^1^Department of Biomedical Engineering, National Taiwan University College of Medicine and College of Engineering, Taipei 100233, Taiwan; ^2^Institute of Biomedical Engineering and Nanomedicine, National Health Research Institutes, Miaoli 35053, Taiwan; ^3^MBInsight Technology Corporation, New Taipei City 236658, Taiwan; ^4^Institute of Medical Device and Imaging, National Taiwan University College of Medicine, Taipei 100233, Taiwan

## Abstract

**Purpose:**

We present a novel background tissue phase removing method, called anatomical phase extraction (APE), and to investigate the accuracy of temperature estimation and capability of reducing background artifacts compared with the conventional referenceless methods.

**Methods:**

Susceptibility variance was acquired by subtracting pretreatment baseline images taken at different locations (nine pretreatment baselines are acquired and called *φ*_1_ to *φ*_9_). The susceptibility phase data *φ*_*S*_ was obtained using the Wiener deconvolution algorithm. The background phase data *φ*_*T*_ was isolated by subtracting *φ*_*S*_ from the whole phase data. Finally, *φ*_*T*_ was subtracted from the whole phase data before applying the referenceless method. As a proof of concept, the proposed APE method was performed on ex vivo pork tenderloin and compared with other two referenceless temperature estimation approaches, including reweighted *ℓ*1 referenceless (RW- *ℓ*1) and *ℓ*2 referenceless methods. The proposed APE method was performed with four different baselines combination, namely, (*φ*_1_, *φ*_5_, *φ*_2_, *φ*_4_), (*φ*_3_, *φ*_5_, *φ*_2_, *φ*_6_), (*φ*_7_, *φ*_5_, *φ*_8_, *φ*_4_), and (*φ*_9_, *φ*_5_, *φ*_8_, *φ*_6_), and called APE experiment 1 to 4, respectively. The multibaseline method was used as a standard reference. The mean absolute error (MAE) and two-sample *t*-test analysis in temperature estimation of three regions of interest (ROI) between the multibaseline method and the other three methods, i.e., APE, RW- *ℓ*1, and *ℓ*2, were calculated and compared.

**Results:**

Our results show that the mean temperature errors of the APE method-experiment 1, APE method-experiment 2, APE method-experiment 3, APE method-experiment 4, and RW- *ℓ*1 and *ℓ*2 referenceless method are 1.02°C, 1.04°C, 1.00°C, 1.00°C, 4.75°C, and 13.65°C, respectively. The MAEs of the RW- *ℓ*1 and *ℓ*2 referenceless methods were higher than that of APE method. The APE method showed no significant difference (*p* > 0.05), compared with the multibaseline method.

**Conclusion:**

The present work demonstrates the use of the APE method on referenceless MR thermometry to improve the accuracy of temperature estimation during MRI guided high-intensity focused ultrasound for ablation treatment.

## 1. Introduction

Recently, high-intensity focused ultrasound (HIFU) has received a surge of attention due to its ability to perform ablation or hyperthermia therapy without an incision [1]. HIFU treatment is superior to conventional resection surgery for several reasons, including reduced cost, shorter recovery time, and greater patient treatment acceptance [2]. During HIFU treatment, monitoring the temperature response is important to ensure that the required thermal dose is delivered to the target region while sparing the surrounding healthy tissues [3]. Magnetic resonance imaging (MRI) is well suited for this purpose because of its great sensitivity of temperature measurement and attractive soft-tissue contrast to clearly reveal protein denaturation and lesion formation [4]. Thus, MRI guided HIFU (MRgHIFU) treatment is widely used in several kinds of diseases, including uterine fibroids [5, 6], brain tumors [7], and essential tremor [8].

MR thermometry can be carried out by several kinds of tissue contrasts, such as proton density [9], T1 relaxation time [10], diffusion coefficient of water molecules [11], and proton resonance frequency shift (PRFS) [12, 13]. Of these, the PRFS method is the most widely used approach because of its linear behavior, ease of measurement, and near tissue-type independence [3, 14]. The PRFS method is based on the chemical shift of water protons [12, 15] and utilizes gradient-echo pulse sequences to acquire MR phase images. With this method, one pretreatment phase image is acquired as a baseline and subsequently subtracted from sequentially acquired phase images during heating to obtain a phase difference and compute the thermal mapping image.

In spite of its success, the PRFS method operates under the assumption that temperature variation is the sole contributor to phase variation. However, in practice, there are multiple sources of phase variations beside temperature variation, such as field drift [16], patient motion [17], heterogeneous fat/water distribution [18, 19], cavitation [20], oxygen concentration changes [21], and ultrasound transducer movement [22]. Among these potential error sources, ultrasound transducer movement is the dominant source of bias during MRgHIFU treatment. These error sources can cause misinterpretation of phase variation as temperature elevation, creating a temperature bias. Correction of this temperature bias is essential to avoid ineffective treatment or unexpected denaturation of adjacent healthy tissues.

Several strategies have been proposed to overcome this issue. A typical method is the multibaseline method, which acquires multiple baseline images to form a lookup table and obtains the corresponding image for baseline subtraction during heating, at the expense of a prolonged scan time [23, 24]. Instead of acquiring multiple baseline images, Rieke et al. proposed a *ℓ*2 referenceless method which acquires baseline images by applying a two-dimensional polynomial fitting of the nonheated region [25], and Grissom et al. introduced a reweighted *ℓ*1 regression to this approach to enhance its convenience (hereafter referred to as the RW-*ℓ*1 referenceless method) [26]. However, tissue-inhomogeneity may cause background artifacts in the temperature maps of both referenceless methods, leading to misjudgment of the focal zone position. These artifacts limit the use of the referenceless methods in clinical applications.

In this study, we introduced an anatomical phase extraction (APE) method to the referenceless MR thermometry whereby the background tissue phase data was isolated and removed before applying polynomial fitting. The APE method was designed to eliminate the detrimental effects of tissue-inhomogeneity. The performance of APE method was evaluated in ex vivo pork tenderloin by using the multibaseline method as standard reference and comparing with the conventional referenceless methods, including *ℓ*2 and RW-*ℓ*1.

## 2. Materials and Methods

### 2.1. MRgHIFU System Setup

The MRgHIFU system design and its experimental setup are shown in Figures 1(a) and 1(b). A spherical HIFU-transducer (focal length: 12 cm, aperture radius: 8 cm, and operating frequency: 1.2 MHz) was mounted on an arc structure attached to the MRI patient table. A water bag filled the space between the HIFU transducer and the object to be ablated. The ultrasound power attenuation through the water bag to the ablated object was less than 1.5%. The MR-compatible arc structure can house mechanical mechanisms and associated devices, providing positional control along two degrees of freedom in an in-plane coordinate system. System software was developed with C and JAVA programming language and supported the necessary functions to perform MRgHIFU ablation procedures such as treatment plan, treatment execution with power and positioning controls, workstation-to-MRI scanner communication, target localization, temperature measurement, and ablated tissue necrosis monitoring. Although the fiber optic thermocouple is a common ground truth used to validate MR thermometry, the HIFU transmission would lead to temperature bias of fiber optic thermocouple measurement surrounding the focal region. Therefore, in this study, we did not measure exact temperature changes using the thermocouple device. Since our purpose was to develop a referenceless method which can provide the similar performance as the conventional method, we chose the multibaseline method as the reference standard.

### 2.2. *Ex Vivo* Experiments

*Ex vivo* pork tenderloin was used in this experiment. Nine HIFU ablations with varying power were conducted in different areas of the pork tenderloin (detailed spatial locations and power are given in Table 1) to simulate susceptibility variances caused by device repositioning in the clinical setting. The porcine specimen was obtained 2 hours before the ex vivo MR experiment and kept under the room temperature in the scan room. The positioning of experimental setup and anatomical localization scan took approximately 20 minutes, and the scan time for temperature mapping was approximately 18.5 minutes (1112 seconds). Thus, the total scan time for the whole experiment was approximately 38.5 minutes, and the porcine specimen was kept fresh during the experiment. HIFU energy was transmitted at positions one through nine at *t* = 79, 169, 259, 349, 439, 529, 619, 709, 799 seconds, respectively, for a 30-second ablation and 60-second cooling time. The time series of HIFU ablation is also shown in Figure 1(c). For PRFS MR thermometry, the spoiled gradient echo sequence was implemented in a 1.5T MRI scanner (Symphony, Siemens, Erlangen, Germany) with the following parameters: repetition time (TR) = 37 ms, echo time (TE) = 17.3 ms, flip angle = 18°, acquisition matrix size = 128 × 77, field of view = 256 × 256 mm, slice thickness = 8 mm. The ablation points were preselected, and nine pretreatment baseline images were obtained for the conventional multibaseline thermometry method to acquire standard reference temperature images for comparison (detailed positions are described in Table 1 and relative positions shown in Figure 2(a)). The APE method has to choose four of these baselines to isolate the background tissue phase data. All images were processed and analyzed off-line using MATLAB (R2016b, The MathWorks, Inc, Natick, MA, USA).

### 2.3. Principle

Let *φ*_*j*_ refer to the baseline phase image data when the moving objects (including the HIFU transducer, MRI RF coil, and water bag in our case) are at position *j*, we adopted three assumption for the APE method.

**Assumption 1 .**

During point-by-point ablation in MRgHIFU, only two kinds of phase signals exist in the baseline phase data: the background tissue phase data from the fixed object, hereafter called *φ*_*T*,*j*_, and the susceptibility phase data from moving objects (including the HIFU transducer, MRI RF coil, and water bag in our case), hereafter called *φ*_*S*,*j*_. Thus, the baseline phase image data, *φ*_*j*_, can be expressed as follows:

(1) $$\begin{array}{c} \varphi_{j}=\varphi_{T,j}+\varphi_{S,j}. \end{array}$$

**Assumption 2 .**

When the moving objects are repositioned to different locations, *φ*_*S*_ is merely translated in the *x* and *z* directions, and the magnitude of *φ*_*S*_ does not change. As for *φ*_*T*_, both magnitude and location of *φ*_*T*_ would not be affected by the moving objects repositioning (hence, *φ*_*T*_ is also referred to as the fixed phase data).

**Assumption 3 .**

The deleterious effects of tissue-inhomogeneity which would lead to background artifacts are contained within *φ*_*T*_.

According to Assumption 3, the background artifacts could be circumvented if *φ*_*T*_ can be removed before utilizing the referenceless methods. Thus, the core of the APE method is to isolate and remove *φ*_*T*,*j*_ from whole baseline phase data *φ*_*j*_. To achieve this aim, we have to acquire *φ*_*S*,*j*_ first then *φ*_*T*,*j*_ can be derived from given *φ*_*S*,*j*_ and *φ*_*j*_ in Equation (1).

### 2.4. The Mathematical Model for the Image Degradation Process

To derive *φ*_*S*,*j*_ from baseline images, a mathematical model for the image degradation process was used in the APE procedures. In our cases, susceptibility-shift process results in degradation of original (thermal) image. Image degradation process can be expressed as Equation (2) and detailed derivate in the appendix.

(2) $$\begin{array}{c} \varphi_{S,i}\left(x,z\right)*H_{i-c}\left(x,z\right)=\varphi_{S,i}\left(x,z\right)-\varphi_{S,c}\left(x,z\right), \end{array}$$

where *φ*_*S*,*i*_(*x*, *z*) and *φ*_*S*,*c*_(*x*, *z*) denote the susceptibility phase data from moving objects when the moving objects are at position *i* and *c*, respectively. The distance between position *i* and *c* can be expressed as ∆*x* and ∆*z* (unit: pixel) along *x* and *z* directions, respectively. *H*_*i*−*c*_ (*x*, *z*) is point spread function (PSF) recording the devices shift effect between *φ*_*i*_ and *φ*_*c*_ (the matrix *H*_*i*−*c*_ (*x*, *z*) can also be considered as degrading operation), and the asterisk symbol (∗) indicates a two-dimensional spatial convolution. As *H*_*i*−*c*_(*x*, *z*) and “*φ*_*S*,*i*_(*x*, *z*) − *φ*_*S*,*c*_(*x*, *z*)” are known (detailed in next section), Equation (2) could be cast as a deconvolution problem, and the Wiener deconvolution method can be used to acquire *φ*_*S*,*i*_(*x*, *z*).

### 2.5. Acquisition of *φ*_*S*,*i*_(*x*, *z*)

#### 2.5.1. PSF (*H*_*i*−*c*_) Established

*H*_*i*−*c*_ is a *N*_*x*_ × *N*_*z*_ matrix recording the device shift effect between *φ*_*i*_ and *φ*_*c*_. In the case of the transducer translated Shift *X*_*i*−*c*_(mm) and Shift *Z*_*i*−*c*_ (mm) in *x* direction and *z* direction, respectively, definition of *H*_*i*−*c*_ is

(3) $$\begin{array}{c} H_{i-c}=\left[h_{kl}\right], \end{array}$$

(4) $$\begin{array}{c} h_{kl}\left\{\begin{array}{cc} 1 & \text{if }\left(k,l\right)=\left(0,0\right),\\ -1 & \text{if }\left(k,l\right)=\left(∆x,∆z\right),\\ 0 & \text{otherwise}, \end{array}\right. \end{array}$$

(5) $$\begin{array}{c} ∆x=\frac{\text{Shift }X_{i-c}}{\left({\text{FOV}}_{x}/N_{x}\right)}, \end{array}$$

where the unit of ∆*x* and ∆*z* is pixel.

#### 2.5.2. Acquisition of “*φ*_*S*,*i*_(*x*, *z*) − *φ*_*S*,*c*_(*x*, *z*)” Term

Recall that *φ*_*i*_ and *φ*_*c*_ refer to the baseline phase image data when the moving objects are at position *i* and *c*, respectively. *φ*_*i*_ and *φ*_*c*_ can be expressed as

(6) $$\begin{array}{c} \varphi_{i}\left(x,z\right)=\varphi_{T,i}\left(x,z\right)+\varphi_{S,i}\left(x,z\right),\\ \varphi_{c}\left(x,z\right)=\varphi_{T,c}\left(x,z\right)+\varphi_{S,c}\left(x,z\right). \end{array}$$

As mentioned previously, *φ*_*T*_ is the fixed phase signal, so theoretically *φ*_*T*,*i*_ should equal *φ*_*T*,*c*_ and *φ*_*T*,*i*_(*x*, *z*) − *φ*_*T*,*c*_(*x*, *z*) = 0. Thus, “*φ*_*S*,*i*_(*x*, *z*) − *φ*_*S*,*c*_(*x*, *z*)” term can be obtained by

(7) $$\begin{array}{c} \varphi_{i}\left(x,z\right)-\varphi_{c}\left(x,z\right)=\left(\varphi_{T,i}\left(x,z\right)+\varphi_{S,i}\left(x,z\right)\right)-\left(\varphi_{T,c}\left(x,z\right)+\varphi_{S,c}\left(x,z\right)\right)=\left(\varphi_{T,i}\left(x,z\right)-\varphi_{T,c}\left(x,z\right)\right)+\left(\varphi_{S,i}\left(x,z\right)-\varphi_{S,c}\left(x,z\right)\right)=0+\left(\varphi_{S,i}\left(x,z\right)-\varphi_{S,c}\left(x,z\right)\right)=\varphi_{S,i}\left(x,z\right)-\varphi_{S,c}\left(x,z\right). \end{array}$$

In other words, “*φ*_*S*,*i*_(*x*, *z*) − *φ*_*S*,*c*_(*x*, *z*)” term can be acquired by just subtracting two baseline images.

#### 2.5.3. Using Wiener Deconvolution Method to Acquire *φ*_*S*,*i*_

Finally, we perform Wiener deconvolution [27] on Equation (2) to obtain *φ*_*S*,*i*_(*x*, *z*) as follows:

(8) $$\begin{array}{c} \varphi_{S,i}\left(x,z\right)\approx {\text{FT}}^{-1}\left(\frac{\text{FT}\left(\varphi_{S,i}\left(x,z\right)-\varphi_{S,c}\left(x,z\right)\right)}{F\left(H_{i-c}\right)}∙\frac{{\left|\text{FT}\left(H_{i-c}\right)\right|}^{2}}{{\left|\text{FT}\left(H_{i-c}\right)\right|}^{2}+K}\right), \end{array}$$

where FT and FT^−1^ mean the two-dimensional Fourier transform and inverse Fourier transform, respectively. *K* is a specified constant acting as a free parameter for optimizing the result.

### 2.6. Phase Unwrapping

All images underwent phase unwrapping prior to the APE method. We used Bruce Spottiswoode's code from the MATLAB Central File Exchange [28], based on the algorithm proposed by Ghiglia et al. [29].

### 2.7. APE Procedures

The procedures of the APE method are displayed in a flowchart of Figure 3 and are described below.

1. Pretreatment phase images, *φ*_*i*_(*x*, *z*), *φ*_*c*_(*x*, *z*), *φ*_*m*_(*x*, *z*), and *φ*_*n*_(*x*, *z*), were acquired where the moving objects were positioned in four different locations
2. With *φ*_*i*_(*x*, *z*) and  *φ*_*c*_(*x*, z), *φ*_*S*,*i*_(*x*, *z*) is derived according to Acquisition of *φ*_*S*,*i*_(*x*, *z*) described above
3. According to Assumption 1, the background tissue phase *φ*_*T*,*i*_(*x*, *z*) caused by the fixed object was isolated by subtracting *φ*_*S*,*i*_(*x*, *z*) from *φ*_*i*_(*x*, *z*)
4. To address the noises, *φ*_*T*,*i*_(*x*, *z*) was subtracted from *φ*_*i*_(*x*, *z*), *φ*_*c*_(*x*, *z*), *φ*_*m*_(*x*, *z*), and *φ*_*n*_(*x, z*), respectively, to acquire *φ*_*S*,*i*_(*x*, *z*), *φ*_*S*,*c*_(*x*, *z*), *φ*_*S*,*m*_(*x*, *z*), and *φ*_*S*,*n*_(*x*, *z*). According to Assumption 2, we know that the magnitude of these four susceptibility phase data are equivalent, and there are merely translated in *x* and *z* directions. Thus, these four susceptibility phase data were all shifted to the location *i* and taking the mean as following equation to alleviate the noises

(9) $$\begin{array}{c} \varphi_{S,i\left(\text{final}\right)}\left(x,z\right)=\frac{1}{4}\left[\varphi_{S,i}\left(x,z\right)+\varphi_{S,c}\left(x-∆x,z-∆z\right)+\varphi_{S,m}\left(x-∆x,z\right)+\varphi_{S,n}\left(x,z-∆z\right)\right]. \end{array}$$

(5) Finally, we subtract *φ*_*S*,*i*(final)_ from *φ*_*i*_ to isolate the fixed phase data, called *φ*_*T*,*i*(final)_

### 2.8. Conversion to Temperature

By introducing Assumption 1 that MR phase data acquired during ablation, *φ*_*j*(*ab*)_, is comprised of two kinds of phase signals, *φ*_*T*,*j*(*ab*)_ and *φ*_*S*,*j*(*ab*)_, into the PRFS equation proposed by Ishihara et al. [7], we calculated temperature change as follows:

(10) $$\begin{array}{c} \varphi_{j\left(ab\right)}=\varphi_{T,j\left(ab\right)}+\varphi_{S,j\left(ab\right),}\\ \Delta T=\frac{\varphi_{j\left(ab\right)}-\varphi_{j}}{\gamma \alpha B_{0}TE}=\frac{\left(\varphi_{T,j\left(ab\right)}+\varphi_{S,j\left(ab\right)}\right)-\left(\varphi_{T,j}+\varphi_{S,j}\right)}{\gamma \alpha B_{0}TE}, \end{array}$$

where *γ* is the gyromagnetic ratio, *α* (−0.01 ppm/°C) is the temperature-dependent coefficient for tissue, *B*_0_ is the amplitude of the static magnetic field, *φ*_*j*(*ab*)_ is the phase data acquired during ablation (comprised of *φ*_*T*,*j*(*ab*)_ and *φ*_*S*,*j*(*ab*)_), and *φ*_*j*_ is the baseline phase data corresponding to *φ*_*j*(*ab*)_. As mentioned previously, *φ*_*T*_ is the fixed phase signal, so theoretically *φ*_*T*,*j*(*ab*)_ should equal *φ*_*T*,*j*_. Thus, the equation can be simplified as follows:

(11) $$\begin{array}{c} \Delta T=\frac{\varphi_{S,j\left(ab\right)}-\varphi_{S,j}}{\gamma \alpha B_{0}TE}. \end{array}$$

To acquire the baseline *φ*_*S*,*j*_, we applied a fourth-order RW-*ℓ*1 referenceless method to *φ*_*S*,*j*(*ab*)_ to remove phase variance in *φ*_*S*,*j*(*ab*)_ due to temperature elevation. Then, temperature map can be obtained from Equation (11) with *φ*_*S*,*j*(*ab*)_ and  *φ*_*S*,*j*_. Note that we applied a fourth-order RW-*ℓ*1 referenceless method to *φ*_*S*,*j*(*ab*)_ to remove phase variance. This step would substantially reduce noise and computational errors generated by the Wiener deconvolution.

### 2.9. Validation of APE Method

To compare the performance of the APE method with other referenceless methods, we derived the temperature maps by using the APE method, multibaseline method, RW-*ℓ*1 [26], and *ℓ*2 referenceless method [25]. We used the code provided by Grissom et al. [22] for the RW-*ℓ*1 referenceless method and the APE method with fourth-order fitting in our data. Based on Rieke et al.'s recommendation [21], we also used fourth-order polynomial fitting in the *ℓ*2 referenceless method. Our APE method modified the RW-*ℓ*1 referenceless method by removing *φ*_*T*_ prior to polynomial fitting. We applied four different baseline combination sets to perform APE method. Let baselines which used in APE method as *φ*_*i*_, *φ*_*c*_, *φ*_*m*_, and *φ*_*n*_. The four baseline combinations sets are (*i*, *m*, *n*, *c*) = (1, 5, 2, 4), (3, 5, 2, 6), (7, 5, 8, 4), and (9, 5, 8, 6) used in APE experiment 1, APE experiment 2, APE experiment 3, and APE experiment 4, respectively. Since our purpose was to develop a referenceless method which can provide the similar performance as the conventional method, we chose the multibaseline method as the reference standard. The accuracy of each MR thermometry map was estimated using the temperature map obtained via the multibaseline method.

To visualize the errors in temperature estimation, we subtracted the multibaseline method temperature map from the temperature maps obtained from the other three methods (APE and RW- *ℓ*1 and *ℓ*2 referenceless methods). Furthermore, to evaluate the temperature measurement errors of the three methods compared to the multibaseline method, we drew three rectangular regions-of-interest (ROI) and calculated the mean absolute temperature difference (or mean absolute error (MAE)) of each ROI. Two-sample *t*-test was performed to investigate the difference of the mean temperature values of ROIs between standard reference and each method. To examine the reproducibility of APE method, we also calculated the MAEs of each ROI of four APE experiments, respectively. Furthermore, we showed the representative temperature maps derived from these experiments and subtracted the temperature map obtained via experiment 1, experiment 2, experiment 3, experiment 4 from experiment 2, experiment 4, experiment 1, and experiment 3, respectively, to visualize the difference between the temperature maps acquired from these experiments.

## 3. Results and Discussion

### 3.1. Results

Susceptibility phase data *φ*_*S*_, which is caused by the moving objects at different positions and derived from the APE method outlined above, is shown in Figure 2(b). The *φ*_*S*_ shift, or susceptibility variance, can be visualized by comparing the contours of the central, or reference, position *φ*_*S*,5_ (in red) with the contours of other positions *φ*_*S*,*i*_ (in blue). Although the variance seems nonsignificant, this susceptibility variance would nevertheless result in noticeable and clinically relevant errors in temperature measurement.  Figure 2(c) shows the susceptibility phase data, *φ*_*S*,2_, and the background tissue phase data, *φ*_*T*,2_, which is separated from whole phase data *φ*_2_. The tissue-inhomogeneity contained in *φ*_2_ and *φ*_*T*,2_ is obviously observed, whereas the remaining *φ*_*S*,2_ becomes much smoother.

The ROI surrounding the ablation points (ROI_1_ and ROI_2_) and the background (ROI_3_) are shown in Figure 4(a). Each ROI contains 12 pixels. The absolute errors in temperature measurement of the 12 pixels within each ROI were averaged to obtain the MAE of each ROI. A total of 230 frames were captured for each ROI, and the MAEs of these frames for each ROI of each method are plotted in Figures 4(b)–4(g). The mean temperature error was derived by averaging all the MAEs (Table 2). The root mean square errors (RMSEs) between multibaseline method and the other methods of each ROI are also shown in Table 2 to compare the performance of each method. The mean temperature errors of the APE method-experiment 1, APE method-experiment 2, APE method-experiment 3, APE method-experiment 4, and RW- *ℓ*1 and *ℓ*2 referenceless method are 1.02°C, 1.04°C, 1.00°C, 1.00°C, 4.75°C, and 13.65°C, respectively. The MAEs and RMSEs of the RW- *ℓ*1 and *ℓ*2 referenceless method were higher than APE experiments, especially in ROI_3_ where the proposed APE method achieved the lowest MAEs and RMSEs of mostly less than 1°C. As compared with multibaseline method, both RW- *ℓ*1 and *ℓ*2 referenceless methods showed significant difference (*p* < 0.05). On the contrary, there was no significant difference between multibaseline method and each APE experiment (*p* > 0.05).

Figures 5(a)–5(d) show the temperature maps derived from the multibaseline, proposed APE, RW-*ℓ*1, and *ℓ*2 referenceless thermometry methods, respectively.  Figure 5(e) shows spatial profiles through the heated area of the respective temperature maps. The multibaseline and proposed APE methods demonstrated considerable similarity in both the temperature map and the spatial profile. On the contrary, the *ℓ*2 method resulted in substantial background artifacts and noticeable discrepancies in both the temperature map and the spatial profile when compared to the multibaseline method. Although the RW- *ℓ*1 method performed better than the *ℓ*2 method, background artifacts were still remarkable.

To visualize the error in temperature measurement of each method, Figure 6 shows the representative difference in temperature maps acquired by subtracting the temperature map obtained via each method (APE, RW- *ℓ*1, and *ℓ*2 referenceless) from the multibaseline temperature map. The difference map of APE method exhibited negligible errors. In contrast, both RW-*ℓ*1 and *ℓ*2 referenceless methods resulted in noticeable background artifacts in the difference map, with the *ℓ*2 method demonstrating the largest background artifacts. The background artifacts of the RW- *ℓ*1 method were still notable, despite being smaller compared to the *ℓ*2 method.

To validate the reproducibility of APE method, Figure 7 shows the representative temperature map of APE experiments 1 to 4. It is obvious that these temperature maps demonstrate considerable similarity, and the noises in their difference maps are negligible. Note that the color bar range of difference maps in Figure 7 has been narrowed to 1°C to 4°C because the difference values are too small to identify.

### 3.2. Discussion

The APE method improves upon the referenceless thermometry methods by eliminating background artifacts and temperature measurement errors in the heated region caused by tissue-inhomogeneity. By removing the background tissue phase data *φ*_*T*_ before implementing the referenceless methods, we reduced the adverse effects of tissue-inhomogeneity and obtained a temperature map comparable to that of the multibaseline method. Moreover, by requiring only four pretreatment baseline images instead of an entire baseline library required by the multibaseline method, our proposed APE method could potentially reduce scan time and improve patient comfortability.

Theoretically, baselines of different methods should be compared with that of the multibaseline method to determine the accuracy of each method. However, our APE method acquires a different baseline compared to other thermometry methods. Generally, baselines comprise of both *φ*_*S*_ and *φ*_*T*_ regardless of whether they were acquired via scanning or polynomial fitting. Our strategy removes *φ*_*T*_ to resolve the undesirable consequences of tissue-inhomogeneity; thus, our baseline and floating images do not contain *φ*_*T*_. Therefore, comparing baselines to determine the accuracy of each thermometry method is not feasible in our case. Instead, to assess the accuracy of each method, we qualitatively compared the temperature maps obtained by each method and quantified the temperature measurement errors by calculating the MAEs.

Repositioning of the moving objects results in shifts in *φ*_*S*_ or susceptibility variation. Susceptibility variation in point-by-point ablation (also referred to as sequential sonications) causes errors in temperature measurement in the PRFS method. To our knowledge, *φ*_*T*_ and *φ*_*S*_ always coexist in phase data and are difficult to distinguish. In this study, we developed a method to separate these two phase sources and remove *φ*_*T*_ from whole phase data, thereby visualizing *φ*_*S*_. Consistent with Assumption 2, our results indicate that when the moving objects are repositioned to different locations, the magnitude of *φ*_*S*_ does not change; rather, *φ*_*S*_ is merely translated in the *x* and *z* directions.

Although both RW- *ℓ*1 and *ℓ*2 referenceless methods suffer from negative effects of tissue-inhomogeneity, tissue-inhomogeneity has a smaller influence on the RW- *ℓ*1 method with regard to the area of the background artifact. The RW- *ℓ*1 method optimizes the *ℓ*2 referenceless method by automatically excluding the heated pixels and noise from the polynomial fitting procedure. This may have partially alleviated the effects of tissue-inhomogeneity by unintentionally excluding some, but not all, pixels affected by tissue-inhomogeneity. Despite the improvements of the RW- *ℓ*1 method, background artifacts and temperature measurement errors are still nonnegligible, limiting its clinical applications. Thus, *φ*_*T*_ isolation and removal are still necessary.

Theoretically, our APE algorithm can separate *φ*_*S*_ and *φ*_*T*_ using any two baselines. However, we found that *φ*_*S*_ would slightly deform along the shift direction, resulting in small inconsistencies in *φ*_*T*_, which should be fixed. To address this problem and diminish noise, we take the mean of *φ*_*S*,*i*_(*x*, *z*), *φ*_*S*,*c*_(*x*−∆*x*, *z*−∆*z*), *φ*_*S*,*m*_(x−∆*x*, *z*), and *φ*_*S*,*n*_(*x*, *z*−∆*z*) to acquire *φ*_*S*,*i*(final)_(*x*, *z*) (as mentioned in APE Procedures' step 4) and then subtract *φ*_*S*,*i*(final)_(*x*, *z*) from *φ*_*i*_(*x*, *z*) to acquire the fixed phase data *φ*_*T*,*i*(final)_.

Our study has some limitations. First, the proposed APE method was developed for two-dimensional susceptibility movement, whereas it is not suitable for susceptibility shifts in three dimensions or cylindrical directions. Thus, it is not viable in three-dimensional or cylindrical positioning devices. Currently, the transducers are typically repositioned along two dimensions (e.g., *x*-*z* directions) in most HIFU ablation treatments, so the proposed APE method is applicable for most of clinical use. In further study, it would be beneficial to improve the proposed APE method to a three-dimensional algorithm for providing more clinical feasibility. Second, the shift of moving objects should be detected when the APE method is performed, but there is not a well-established method to detect these shifts to the best of our knowledge. Thus, it is necessary to develop an approach to record the moving objects shifts in MRgHIFU treatment for strengthening its further clinical use.

This study described an APE method which reduces the effect of tissue-inhomogeneity on referenceless methods and improve the accuracy of PRFS-based temperature measurement. This strategy expands the potential clinical applications of the referenceless methods to beyond homogenous tissues. With our APE method, the referenceless methods can potentially be used in clinical MRgHIFU treatment. Compared to the conventional multibaseline method, the APE method demonstrates comparable accuracy and not only avoids unnecessary risk of treatment interruptions arising from patient movements but also decreases preparation time spent obtaining baseline images. Further studies applying the APE method to *in vivo* experiments are necessary to validate its feasibility.

## 4. Conclusion

In this work, we proposed the APE method, a strategy to eliminate the detrimental consequences of tissue-inhomogeneity in referenceless methods. The theoretical aspects of the strategy were described, and an ex vivo experiment was performed for qualitative and quantitative evaluation. Our results indicate that the accuracy of the APE method is comparable with the conventional multibaseline method, implying that the APE method could potentially reduce the total scan time, thereby improving patient comfortability and further reducing the risk of treatment interruption.

## Figures and Tables

**Figure 1:** (a) Schematics and (b) photograph of experimental setup. Spherical HIFU-transducer was mounted on an arc structure attached to the MRI patient table. A water bag filled the space between the HIFU transducer and the object to be ablated. (c) *Ex vivo* experiments with pork tenderloin: ultrasound transducer performed ablation in nine different positions. Upper row: the time series of HIFU ablation. Lower row: the representative temperature maps of the nine ablation positions with the corresponding time. Note that HIFU ablation power transmitted in nine different positions was varying and increasing (detailed in Table 1), and thus, the temperature of successive points becomes hotter and hotter.

**Figure 2:** (a) Schematic diagram of relative positions one through nine. The distance between adjacent points is 10 mm. (b) Susceptibility phase signal images at the nine different positions acquired by the APE method. The contour of the central, or reference, position *φ*_*S*,5_ (in red) is superimposed on each susceptibility phase signal image to visualize the susceptibility variance between different positions. (c) Representative whole phase data (*φ*_2_), background tissue phase data (*φ*_*T*,2_), and susceptibility phase data (*φ*_*S*,2_). The tissue-inhomogeneity of *φ*_*T*,2_ is apparent. When *φ*_*T*,2_ is removed from *φ*_2_, the remaining *φ*_*S*,2_ is smooth.

**Figure 3:** Flowchart of APE procedures. *φ*_*i*_: baseline phase image when the moving objects are at position *i* (note that *φ*_*i*_ = *φ*_*S*,*i*_ + *φ*_*T*,*i*_); matrix *H*_*i*−*c*_: records the effect of *φ*_*S*,*i*_ − *φ*_*S*,*c*_; *φ*_*S*,*i*_ − *φ*_*S*,*c*_: equals the convolution of (*φ*_*S*,*i*_, *H*_*i*−*c*_); *φ*_*S*,*i*_: susceptibility phase signal when the moving objects are at position *i*; *φ*_*T*,*i*_: background tissue phase signal when the moving objects are at position *i*.

**Figure 4:** (a) A representative temperature map with the three selected ROIs. Each ROI contains 12 pixels, and the absolute errors in temperature measurement of the 12 pixels within each ROI were averaged to obtain the MAE. (b–g) The MAEs of a total of 230 frames among these three ROIs for the proposed APE #experiment 1 (b), proposed APE #experiment 2 (c), proposed APE #experiment 3 (e), proposed APE #experiment 4 (f), and RW- *ℓ*1 (d) and *ℓ*2 referenceless (g) methods, respectively.

**Figure 5:** Temperature maps derived from the (a) multibaseline, (b) proposed APE, (c) RW-*ℓ*1 referenceless, and (d) *ℓ*2 referenceless method, respectively. (e) Comparison of spatial profiles through the heated area (dotted-white line) derived from (a) to (d).

**Figure 6:** (a) Temperature maps derived from the multibaseline (standard reference) method. (b) Temperature maps derived from the proposed APE (top row), RW- *ℓ*1 referenceless (middle row), and *ℓ*2 referenceless (bottom row) methods. (c) The difference between temperature maps of the multibaseline method and the other three methods. Background artifacts in the RW- *ℓ*1 referenceless and *ℓ*2 referenceless methods are strikingly obvious. The proposed APE method markedly reduced these background artifacts.

**Figure 7:** The representative temperature map of APE experiments 1 to 4 and the difference map acquired from temperature map difference of experiment 1-experiment 2, experiment 2-experiment 3, experiment 3-experiment 4, and experiment 1-experiment 4. It is obvious that these temperature maps demonstrate considerable similarity, and the noises in their different maps are negligible.

**Table 1:** *Ex vivo* HIFU ablation parameters.

Location	Coordinate (*x*, *z*)	Shift *X* (mm)	Shift *Z* (mm)	HIFU power^a^ (W)
1	(10, 10)	10	10	40
2	(0, 10)	0	10	60
3	(-10, 10)	10	10	80
4	(10, 0)	10	0	100
5	(0, 0)	0	0	120
6	(-10, 0)	10	0	140
7	(10, -10)	10	10	160
8	(0, -10)	0	10	180
9	(-10, -10)	10	10	200

^a^Ablation duration: 30 seconds; cooling interval: 60 seconds.

**Table 2:** Mean values and standard deviations for absolute temperature estimation errors, RMSEs, and two-sample *t*-test analysis between multibaseline and proposed APE, RW − *ℓ*1 referenceless, and *ℓ*2 referenceless method, respectively.

	ROI_1_	ROI_2_	ROI_3_	*p* value
Proposed APE (°C)				
#experiment 1	1.14 ± 0.69 (RMSE = 1.33)	1.08 ± 1.04 (RMSE = 1.50)	0.83 ± 0.37 (RMSE = 0.90)	0.35
#experiment 2	1.15 ± 0.68 (RMSE = 1.33)	1.11 ± 1.07 (RMSE = 1.53)	0.88 ± 0.37 (RMSE = 0.95)	0.40
#experiment 3	1.17 ± 0.69 (RMSE = 1.36)	0.96 ± 0.91 (RMSE = 1.32)	0.86 ± 0.38 (RMSE = 0.94)	0.41
#experiment 4	1.14 ± 0.69 (RMSE = 1.34)	1.06 ± 1.02 (RMSE = 1.47)	0.79 ± 0.35 (RMSE = 0.87)	0.32
RW-*ℓ*1 referenceless (°C)	1.37 ± 0.84 (RMSE = 1.61)	3.00 ± 0.37 (RMSE = 3.03)	9.89 ± 0.98 (RMSE = 9.93)	< 0.05
*ℓ*2 referenceless (°C)	2.76 ± 0.78 (RMSE = 2.86)	1.98 ± 1.49 (RMSE = 2.48)	36.20 ± 1.34 (RMSE = 36.22)	< 0.05

## Data Availability

The data used to support the findings of this study are available from the first author (d06548024@ntu.edu.tw) upon request.

## Appendix

### A. Derivation of Equation (2)

From definition of two-dimensional convolution, the left side of Equation (2) is

(A.1) $$\begin{array}{c} \varphi_{S,i}\left(x,z\right)*H_{i-c}\left(x,z\right)=\overset{M-1}{\underset{m=0}{\sum }}\overset{N-1}{\underset{n=0}{\sum }}\varphi_{S,i}\left(x,z\right)\;H_{i-c}\left(m-x,n-z\right). \end{array}$$

From Equation (4), we can see that *H*_*i*−*c*_(*m* − *x*, *n* − *z*) would be nonzero only if

(A.2) $$\begin{array}{c} \left\{\begin{array}{c} m-x=0,\\ n-z=0, \end{array}\right. \end{array}$$

and

(A.3) $$\begin{array}{c} \left\{\begin{array}{c} m-x=∆x,\\ n-z=∆z. \end{array}\right. \end{array}$$

Thus, Equation (A.1) can be rewritten as follows:

(A.4) $$\begin{array}{c} \varphi_{S,i}\left(\text{x},\text{z}\right)*H_{i-c}=\varphi_{S,i}\left(m,n\right)\;H_{i-c}\left(1,1\right)+\varphi_{S,i}\left(m-∆x,n-∆z\right)\;H_{i-c}\left(∆x,∆y\right). \end{array}$$

According to Equation (4)

(A.5) $$\begin{array}{c} \;H_{i-c}\left(1,1\right)=1,\\ \;H_{i-c}\left(∆x,∆y\right)=-1. \end{array}$$

Equation (A.4) can be equivalently expressed as

(A.6) $$\begin{array}{c} \varphi_{S,i}\left(x,z\right)*H_{i-c}\left(x,z\right)=\varphi_{S,i}\left(m,n\right)-\varphi_{S,i}\left(m-∆x,n-∆z\right). \end{array}$$

According to Assumption 2, *φ*_*S*,*i*_ is merely a translation of *φ*_*S*,*c*_, and ∆*x* and ∆*z* represent the shift distance along *x* and *z* directions between *φ*_*S*,*i*_ and *φ*_*S*,*c*_. Thus, making the substitution *φ*_*S*,*c*_ = *φ*_*S*,*i*_(*m*−∆*x*, *n*−∆*z*) gives

(A.7) $$\begin{array}{c} \varphi_{S,i}\left(x,z\right)*H_{i-c}\left(x,z\right)=\varphi_{S,i}\left(x,z\right)-\varphi_{S,c}\left(x,z\right). \end{array}$$

Hence, Equation (2) is proved.
